This article has been retracted.

# Evaluation of Therapeutic Effect and Prognosis of Danzhi Xiaoyao Powder Combined with Photodynamic Therapy in the Treatment of Rose Acne

**DOI:** 10.1155/2022/1636839

**Published:** 2022-03-11

**Authors:** Xinjian Yu, Ni Zhang, Jing Jin, Xuwen Yin, Jing Luo

**Affiliations:** ^1^Hubei Provincial Hospital of Traditional Chinese Medicine, Dermatological Department, Attending Psychiatrist, 430061, China; ^2^Hubei Provincial Hospital of Traditional Chinese Medicine, Dermatological Department, Supervising Technician, 430061, China

## Abstract

**Background:**

Rose acne is a chronic inflammatory skin disease that can cause paroxysmal flushing, persistent erythema, papules or papules on the face, and pustules, and it has a greater impact on the life of patients, so it is important to treat it.

**Objective:**

To investigate the effect of Danzhi Xiaoyao Powder combined with photodynamic therapy (PDT) on the curative effect evaluation and prognosis of patients with rose acne. *Patients and Methods*. The clinical data of 110 rose acne patients who were treated in our hospital from January 2019 to January 2021 were selected as the subject of this retrospective study. They were divided into a control group and a treatment group according to the random residue grouping method. The new crown epidemic, loss to follow-up, etc. fell out of 5 cases in each group, and finally, 50 cases in each group were left. Among them, the control group was treated with PDT, and the treatment group was combined with Danzhi Xiaoyao Powder on the basis of the control group. Then we observe and compare the effects of skin lesion scores and clinical symptom scores and differences in clinical efficacy between the two groups.

**Results:**

The comparison of the clinical symptom scores of the two groups of patients before treatment was not statistically significant (*P* > 0.05), while the burning score, tingling score, dryness score, and pruritus score of the treatment group after treatment were significantly different. The internal comparison after treatment was lower than before treatment, and the comparison between the treatment groups was significantly higher than the control group, which was statistically significant (*P* < 0.05). There was no statistically significant difference in the skin lesion scores of the two groups before treatment (*P* > 0.05), while the papules score, pustule score, erythema score, and telangiectasia score of the treatment group after treatment were significantly different and compared within the group. After treatment, the treatment group was significantly higher than the control group, and the comparison was statistically significant (*P* < 0.05). The effective rate of 98.00% in the treatment group was significantly higher than the 76.00% in the control group, and the difference was statistically significant (*P* < 0.05). The clinical efficacy of the two groups of patients showed that the rash, chest tightness, nausea, and diarrhea of the treatment group were significantly lower than those of the control group, and the difference was statistically significant (*P* < 0.05).

**Conclusion:**

Danzhi Xiaoyao Powder combined with PDT to treat rose acne is effective, can quickly control inflammatory papules and inflammatory erythema, effectively improve the clinical symptoms of patients, and reduce adverse reactions.

## 1. Introduction

Rose acne is a chronic inflammatory skin disease that mainly involves facial blood vessels and hair follicle sebaceous glands. Its rash is manifested as paroxysmal flushing, persistent erythema, telangiectasia, papules, or papulopustular herpes, with or without subjective symptoms such as burning, tingling, dryness, or itching; some patients also have eye symptoms [1]. The etiology of rose acne is unknown. Among them, abnormal natural immune function, abnormal neurovascular regulation, endocrine disorders, microbial infection, genetics, abnormal skin barrier function, and other factors may be its pathogenesis and aggravating factors [2]. At present, there are many treatments for rose acne, including not only topical medications but also oral medications and surgical treatments. However, patients with topical medications have poor compliance and relatively more side effects of oral medications. These treatments have limited effects and can only be controlled and relieved. Some of the patients' symptoms are traumatized by surgery and are not accepted by the patients. Therefore, we began to explore new treatment methods that can achieve the therapeutic effect and be accepted by the patients.

Our research uses photodynamic therapy (PDT), a technology that uses photodynamic effects for disease diagnosis and treatment [3]. The basic principle is that the photosensitizer interacts with molecular oxygen in the surrounding environment under a specific-wavelength laser or light excitation to produce singlet oxygen, which can induce apoptosis and necrosis, vascular damage, inflammation, and immune regulation [4]. As a noninvasive and simple operation and having high safety, fast onset, and less adverse reactions, PDT is more and more popular among patients. It is safe and effective for rose acne and can quickly control inflammatory papules and inflammatory erythema, but it is resistant to paroxysmal rose acne, whose main manifestation is flushing, and has poor efficacy [5]. Danzhi Xiaoyao Powder has the therapeutic effects of soothing the liver and relieving depression, treating liver depression, and transforming fire, hot flashes, and zygomatic redness and has a good effect on the paroxysmal flushes that occur with rose acne [6]. Based on this, our hospital has conducted a certain exploration to explore the curative effect evaluation and prognosis of Danzhi Xiaoyao Powder with PDT in the treatment of rose acne. The current research results are reported as follows.

## 2. Material and Methods

### 2.1. General Information

The study actually included a sample size of 100 cases, which were divided into a control group and a treatment group with 50 cases in accordance with the random remainder grouping method. Chinese medical diagnostic criteria are as follows: All patients meet the diagnostic criteria for rose acne in the “People's Republic of China Traditional Chinese Medicine Industry Standards· Traditional Chinese medicine (TCM) Dermatology Syndrome Diagnostic Efficacy Criteria” [7]. The selected patients' TCM syndromes are all liver-stagnation and blood-heat syndromes. The main symptoms are as follows: Rice grain-sized papules or small pustules can be seen on the basis of persistent erythema on the face, without obvious blackheads. It may be accompanied by a dilatation of capillaries, such as red filaments entwined, and criss-cross, and the skin color changes from bright red to purple-brown, with consciously mild itching. Secondary symptoms are as follows: local skin burning, tingling, dryness, itching, irritability, spontaneous sweating, dry mouth, bitter mouth, irregular menstruation, fullness of the chest and flanks, constipation, yellow urine, and red tongue. The moss is thin and yellow, and the pulse string is several. Medical diagnostic criteria in European and American countries are as follows: All patients meet the diagnostic criteria of rose acne in “Standard classification and pathophysiology of rosacea: The 2017 update by the National Rosacea Society Expert Committee” [8]. The main symptoms are as follows: cheek, perioral, or nose. The obvious cause is paroxysmal flushing, and the flushing is obviously affected by factors such as temperature, mood, and ultraviolet rays, or persistent erythema appears. Secondary symptoms are as follows: (1) skin sensitivity symptoms such as burning, tingling, dryness, or itching; (2) dilation of the cheek or perioral or nasal capillaries; (3) cheek, perioral, or nasal papules or papules; and (4) eye symptoms. We exclude obvious causes such as oral isotretinoin capsules or chemical peels or topical glucocorticoids that cause paroxysmal flushing or persistent erythema caused by damage to the skin barrier. The necessary conditions can be diagnosed by adding and above minor conditions for rose acne. General data such as gender and age of the two groups of patients had no effect on this test, as shown in Table 1.

### 2.2. Inclusion and Exclusion Criteria

Inclusion criteria are as follows: (1) Patients who meet the diagnostic criteria of rose acne and the selected patients' TCM syndromes are all patients with liver-stagnation and blood-heat syndrome, aged 18 to 60 years old; (2) without oral or topical use of retinoic acid in the past three months, or within the past one month, those who have not taken glucocorticoids, anti-infective drugs, and antiallergic drugs and have not used any other methods to treat rose acne; (3) the patient's heart, lung, liver, and kidney functions are basically normal, and there is no important organ disease or hematopoietic system disease. According to researchers, for diseases that are not suitable for participating in clinical trials, the patient's clinical data is complete. Exclusion criteria are as follows: (1) Persons allergic to porphyrins, persons with a history of photosensitivity, topical antibiotics, retinoic acid drugs, glucocorticoids, benzoyl peroxide, and other drugs were treated within one month, had a history of sun exposure in the past month, received photoelectric therapy for three months, or received facial grinding treatment within half a year; (2) patients using vasodilators, *β*-receptor blockers, anticoagulants, and other drugs that affect the symptoms of rose acne, combined with facial acne, atopic dermatitis, hormone-dependent dermatitis, and other facial skin-related diseases; and (3) patients with a history of mental illness, pregnant or lactating women, those planning to become pregnant in the near future, or those with incomplete clinical data.

### 2.3. Method

The control group was treated with PDT, that is, patients were required to avoid direct sunlight during the treatment period, moisturize and protect the face (use medical cosmetics as much as possible), eat lightly, avoid eating spicy irritants and consuming caffeine, avoid exposure to the sun, and limit smoking, wine, etc. Before treatment, the relevant matters were explained to the research subjects, the facial skin was cleaned, Ella was formulated into fresh glue with a concentration of 5%, and the freshly prepared glue was applied on the lesion and the 0.5 c normal skin and mucous membranes around it, with light encapsulation (1~2 hours), and then the face was washed with clean water until the skin is not greasy. The research subjects wear protective goggles and use the LED-IB photodynamic therapy instrument. The output wavelength is 633 ± 10 nm, and localized irradiation was performed. The output power is 60-100 mW/cm^2^, the distance between the lamp and the facial skin lesions is about 10 cm, and the irradiation time is 20 minutes each time. Immediately after treatment, cold spray or cold compress was used for at least 30 minutes. Light was strictly avoided within 48 hours of treatment, and we wait for the scab to fall off naturally for about 1 week. During this period, no makeup, hot bath, or scratching of the treated area is required for once a week, 4 times in total.

The treatment group added Danzhi Xiaoyao Powder addition and subtraction, Di Yin Fang cold compress, and metronidazole gel external application on the basis of the control group, namely Danzhi Xiaoyao Powder (Mudan Peel 10 g, Fried Shanzhi 9 g, Angelica 12 g, White Peony Root 10 g, Bupleurum 6 g, Poria 12 g, Atractylodes 12 g, and Licorice 6 g). If the patient has severe damp-heat and pustules, *Scutellaria baicalensis* Georgi, *Coix* seed, Yinchen, *Poria coix*, and *Polyporus umbellatus* were added to clear away heat and invigorate the spleen and dehumidify; if the patient has internal heat toxins and severe redness and swelling, honeysuckle, dandelion, and purple flowers were added. Ding is used to clear away heat and detoxify; if the patient's lung meridian is wind-heat with severe itching, honeysuckle, purslane, and white fresh skin were added to relieve wind and heat, detoxify, and relieve itching; if the patient's blood heat is full, *Imperata cylindrica* and *Sophora japonicus* were added. The flower, *Rehmannia*, and elm were added to clear the heat and cool the blood. When decocting the medicine, you need to add water 3-5 cm higher than that of traditional Chinese medicine. The amount of water for the second decocting is gradually reduced. The first decocting takes 20-25 min, and the second decocting takes 15-20 min. After decocting, 200 ml of concoction should be filtered out immediately after breakfast, and 100 ml each was taken after dinner. Di Yin Fang is used to apply cold compresses to the skin lesions. The gauze fits closely to the skin lesions, and the size is the same as the affected area. Each application is 30-40 min, 5-10 min change, twice a day. The temperature of the liquid medicine is generally around 10°C. Auxiliary topical 0.75% metronidazole gel (Jiangsu Zhiyuan Pharmaceutical Co., Ltd., Sinopharm H10980213) is applied to the skin lesions in the morning and evening after cleansing. The above treatment was continuously treated for 4 weeks.

### 2.4. Follow-Up and Observation Indicators

Before treatment and at the end of 4 weeks of treatment, the two groups of patients were tested for the effect of clinical symptom scores, skin lesion scores, and clinical efficacy differences. (1) Clinical symptom score is as follows [9]: It mainly includes four items: burning, tingling, dryness, and itching, and each symptom score is 0-3 points; the higher the score, the more obvious the symptoms. (2) Skin lesion score is as follows [10]: It mainly includes four items: erythema, papules, pustules, and telangiectasia, and each symptom score is 0-3 points; the higher the score, the more obvious the skin lesion symptoms. (3) Clinical efficacy is established in accordance with the “Guiding Principles for Clinical Research of New Chinese Medicines (Trial)”): recovery: most or all of the skin lesions disappeared, 70% ≤ symptom score reduction ≤ 100%; improvement: only some skin lesions disappeared, 40% ≤ If the symptom score drops < 70%, which is invalid: the skin lesions are not resolved obviously, and the symptom score drops < 40%. Effective rate = (healed + improved) · 100%.

### 2.5. Statistical Methods

The data in this study was calculated using Excel and reviewed by two physicians. The selected data are in accordance with the normal distribution. After the first author and corresponding author have entered the data into the computer system and proofread, the statistical software is used for SPSS25.0 to perform related calculations. Measurement data were expressed as mean ± standard deviation ($\bar{x}\pm s$) by the independent-sample *t*-test, count data expressed as a percentage (%) or whole number were used by the *χ*^2^ test, and statistical *P* < 0.05 indicated that the difference was statistically significant.

## 3. Results

### 3.1. Demographic Characteristics

The general data of the two groups of patients, such as gender, average age, average course of the disease, weight, and skin lesion location, were not significantly different by the *t*-test and chi-square test (*P* > 0.05). All the data are shown in Table 1.

### 3.2. Comparison of Clinical Symptom Scores

The clinical treatment effect is shown in Figures 1–3. The comparison of the clinical symptom scores of the two groups before treatment was not statistically significant (*P* > 0.05), while the comparison of the burning score, tingling score, dryness score, and pruritus score of the treatment group after treatment was significantly different, and the comparison within the group after treatment was lower than before treatment; the treatment group was significantly higher than the control group, and the comparison was statistically significant (*P* < 0.05). All the data are shown in Table 2.

### 3.3. Comparison of Skin Lesion Scores

There was no statistically significant difference in the skin lesion scores of the two groups before treatment (*P* > 0.05), while the papules score, pustule score, erythema score, and telangiectasia score of the treatment group after treatment were significantly different, and compared within the group, after treatment was lower than before treatment; the treatment group was significantly higher than the control group, and the comparison was statistically significant (*P* < 0.05). All the data are shown in Table 3.

### 3.4. Comparison of Clinical Efficacy and Complications

The effective rate of 98.00% in the treatment group was significantly higher than the 76.00% in the control group, and the difference was statistically significant (*P* < 0.05). The clinical efficacy of the two groups of patients showed that the rash, chest tightness, nausea, and diarrhea of the treatment group were significantly lower than those of the control group, and the difference was statistically significant (*P* < 0.05). All the data are shown in Table 4.

## 4. Discussion

Rose acne tends to occur in women aged 30-50. Facial skin lesions are recurrent and difficult to heal. Long-term facial troubles may lead to depression or anxiety. Rose acne may be triggered by a variety of factors with abnormal activation of natural immunity and vascular function. Abnormality is the dominant chronic inflammatory skin disease, and some patients have family aggregation [11]. In recent years, there have been reports in the literature that PDT of rose acne can significantly improve clinical symptoms, but little is known about the mechanism of PDT in the treatment of rose acne [12]. The mechanism of PDT in the treatment of rose acne is unclear. Its possible mechanisms include the following: using light energy to activate the photodynamic effect, producing singlet oxygen and free radicals and other cytotoxic substances, destroying cell structure and function, and thereby inhibiting excessive sebum secretion and promoting skin lesion healing and other effects [13]. PDT can affect the expression of Toll-like receptors and the secretion of cytokines and affect the secretion of matrix metalloproteinases (MMP) 1 and MMP3 by fibroblasts to regulate the immune system and induce apoptosis of T lymphocytes [14]. Microbes such as *Demodex folliculorum* can synthesize and store a large amount of porphyrin by themselves, promote the photochemical reaction, are directly killed by red light, inhibit the expansion of blood vessels in the dermis, and change the local inflammatory microenvironment by adjusting inflammatory factors [15].

In this study, the difference of burning score, stinging score, dryness score, and itching score of patients in the treatment group after treatment was significantly different and lower than before treatment, while the treatment group was significantly higher than the control group, indicating that rose acne was treated with Danzhi Xiaoyao Powder combined with PDT, which effectively improved the clinical symptoms of patients. The reasons for the analysis are as follows: for patients with rose acne, treatment should be based on draining the liver and relieving depression, clearing heat, and dispersing nodules, and Danzhi Xiaoyao Powder was chosen as the main formula for addition and reduction. In Danzhi Xiaoyao Powder, *Gardenia jasminoides* goes inside and clears internal heat, Mudanpi and Red Peony clear the heat and cool the blood to disperse blood stasis, and raw gypsum clears the actual heat in the Qi part of the lung and stomach [16]. *Scutellaria baicalensis* and Radix et Rhizoma forsythiae clear the heat and detoxify toxins, disperse nodules, and eliminate carbuncles; *Citrus aurantium* broadens the middle and lowering Qi, dissolves phlegm, removes lumpiness, with Chai Hu one ascending and one descending, regulates the Qi flow in the chest, and opens the depression in the chest; *Angelica sinensis* and Radix et Rhizoma nourish blood and Yin and prevent excessive consumption; Hawthorn is sour and enters the liver meridian, eliminates food stagnation, activates blood circulation, disperses stasis, and helps restore the draining function of the liver; it is supplemented with a small amount of *Atractylodes macrocephala*, *Poria*, and *Glycyrrhiza glabra* to strengthen the spleen, in order to “see the disease of the liver. It is also supplemented with a small amount of *Atractylodes macrocephala*, *Poria cocos*, and *Glycyrrhiza glabra* to strengthen the spleen, so that “when we see the disease of the liver, we know that the liver transmits the spleen, so we should first strengthen the spleen” [17]. It is an important treatment for diseases caused by emotional and mental disorders. Some studies have shown that the addition and subtraction of the formula based on Zhuangyao San have the effect of regulating emotions, antidepressants, and regulating neuroendocrine function. Modern pharmacological studies have shown that Chai Hu has hepatoprotective, sedative, anti-inflammatory, and immunomodulatory effects [18]. *Scutellaria baicalensis* and *forsythia* have anti-inflammatory and antiallergic effects, and *B. alba* can enhance the immunity of the body, stimulate the proliferation of reticuloendothelial cells, enhance the phagocytosis of leukocytes, have antibacterial and anti-inflammatory effects, and also have a strong inhibitory effect on the secretion of sebaceous glands and antiandrogenic effects [19]. Tanshinone solid, an extract of the Chinese herbal medicine Salvia miltiorrhiza, has a broad-spectrum antibacterial effect and strong antibacterial activity against *Propionibacterium* acnes, as well as mild estrogen-like activity, antiandrogenic effect, and antisebaceous gland secretion [20]. Currently, it is widely used in the treatment of acne; however, in clinical practice, Danzhi Xiaoyao Powder with psychological detoxification was found to be more effective than Danshinone internally in the treatment of acne with liver meridians and heat, suggesting that psychological detoxification plays a synergistic role in the treatment of acne [21].

In this study, the difference in papule score, pustule score, erythema score, and capillary dilatation score of patients in the treatment group after treatment was significant and lower than before treatment, and significantly higher in the treatment group than in the control group, indicating that rose acne treated with Danzhi Xiaoyao Powder combined with PDT for rose acne can rapidly control inflammatory papules and inflammatory erythema. The specific reasons for this are as follows: According to TCM, the liver is responsible for normal drainage function, the body's Qi and blood are harmonized, and the emotions and spirit are regulated in order to resist the stimulation of the external environment and make adaptive adjustments to avoid disease. At present, Chinese rose acne diagnosis and treatment experts divide rose acne into four types, among which the treatment of liver depression and blood heat evidence is to dredge the liver to relieve depression, clear the heat, cool the blood, and treat skin appendage diseases, such as rose acne, acne, and baldness, as well as treat skin pruritus, neurodermatitis, and other skin diseases related to neuropsychiatric disorders [22]. In TCM, the erythematous phase of rose acne is mild, mostly due to heat in the lung and stomach, or heat that produces wind with acute onset; moderate rose acne patients have persistent erythema, or with papules and pustules, mostly due to liver heat and blood stasis; late skin thickening, as well as nasal redundancy generation, is due to Qi stagnation and blood stasis, and evil toxins are contained within [23]. Rose acne's prolonged and difficult-to-heal clinical characteristics easily affect the patient's spirit and mood, should be treated by the clinical characteristics of rose acne that are difficult to heal tend to affect the patient's spirit and mood, and should be treated from the liver by draining the liver and regulating the Qi and regulating the mood. Stagnation of Qi and blood is an important cause for the occurrence and aggravation of rosacea in modern people [24]. In the treatment, the importance of moving Qi and blood, draining the liver, and relieving depression is particularly emphasized, while attention is paid to the application of heat-clearing and blood-cooling drugs to achieve the effect of clearing heat, cooling blood, activating blood, moving Qi, and relieving depression. PDT is a new therapeutic method using photosensitive drugs and laser activation, which is based on the photodynamic effect, causing functional or morphological changes in cells or biomolecules of the organism. Clinical studies have shown that exogenous 5-aminoketovaleric acid as a photosensitizer, selectively acting in the patient's sebaceous gland units, activated by wavelength light can destroy sebaceous gland cells and inhibit excessive sebaceous gland secretion and is now widely used in nontumor type diseases and disfiguring diseases. PDT has the following points [25]: less invasive, low toxicity, good selective applicability, repeatable treatment, and photodynamic. The kinetic response has no effect on the unirradiated part and hematopoietic function. The elimination of occult lesions can destroy microscopic lesions that cannot be seen by the naked eye, reduce the chance of recurrence, and can protect the patient's appearance and vital organ functions while killing harmful tissues [25].

Although this study has some novelty, it also has shortcomings: in objective evaluation index and subjective evaluation index, laboratory index was not included, the results may be biased, and the clinical efficacy of Danzhi Xiaoyao Powder with PDT treatment on rose acne is significant, but the specific mechanism has not been studied in-depth for a long time. In the treatment, we used skin barrier repair with medical skincare products as the basic treatment but failed to establish a separate control group to evaluate the improvement of skin lesions and subjective symptoms of patients with rose acne by basic treatment.

In conclusion, Danzhi Xiaoyao Powder combined with PDT for the treatment of rose acne is effective in rapidly controlling inflammatory papules and erythema, effectively improving patients' clinical symptoms and reducing adverse reactions, which provides a certain reference value for the treatment of rose acne.

## 5. Conclusion

Danzhi Xiaoyao Powder combined with PDT is significantly better than PDT alone in the treatment of rosacea. It can quickly control inflammatory papules and inflammatory erythema, effectively improve patients' clinical symptoms, and reduce adverse reactions.

## Figures and Tables

**Figure 1:** Therapeutic effect of Danzhi Xiaoyao Powder combined with the photodynamic therapy in the treatment of rose acne on the face.

**Figure 2:** Therapeutic effect of Danzhi Xiaoyao Powder combined with photodynamic therapy in the treatment of rose acne on the left face.

**Figure 3:** Therapeutic effect of Danzhi Xiaoyao Powder combined with photodynamic therapy in the treatment of rose acne on the right face.

**Table 1:** Comparison of general information between the two groups (*n*, $\bar{x}\pm s$).

Group	Gender (male/female)	Average age (age)	Mean disease course (moon)	Weight (kg)	Skin lesions location		
					Cheek	Nose and perinasal area	Other
Control group (50)	10/40	40.18 ± 1.32	23.34 ± 3.25	53.36 ± 2.25	36	8	6
Therapy group (50)	9/41	39.62 ± 2.66	22.91 ± 2.64	53.31 ± 2.51	35	10	5
*χ* ^2^/t	0.065	1.333	0.726	0.105	0.327		
*P*	0.799	0.185	0.469	0.917	0.849		

**Table 2:** Comparison of clinical symptom scores between the two groups ($\bar{x}\pm s$).

Group		Searing score	Tingling score	Dryness score	Pruritus score
Control group (50)	Before treatment	2.28 ± 0.32	1.94 ± 0.25	1.81 ± 0.32	0.21 ± 0.02
	After treatment	1.62 ± 0.16^a^	0.86 ± 0.24^a^	1.05 ± 0.11^a^	0.12 ± 0.03^a^
Therapy group (50)	Before treatment	2.24 ± 10.25	1.91 ± 0.12	1.83 ± 0.27	0.23 ± 0.04
	After treatment	0.61 ± 0.14^ab^	0.37 ± 0.02^ab^	0.24 ± 0.06^ab^	0.06 ± 0.01^ab^

Note: compared with before treatment, ^a^*P* < 0.05. Compared with the control group, ^ab^*P* < 0.05.

**Table 3:** Comparison of skin lesion scores between the two groups ($\bar{x}\pm s$).

Group		Papules score	Pustule score	Erythema score	Telangiectasia score
Control group (50)	Before treatment	5.21 ± 1.23	3.77 ± 0.18	9.04 ± 1.25	4.65 ± 0.82
	After treatment	0.61 ± 0.12^a^	0.87 ± 0.20^a^	4.33 ± 0.24^a^	0.77 ± 0.11^a^
Therapy group (50)	Before treatment	5.13 ± 1.57	3.68 ± 0.26	9.16 ± 1.15	5.02 ± 1.15
	After treatment	2.24 ± 0.53^ab^	2.23 ± 0.26^ab^	1.75 ± 0.26^ab^	2.33 ± 0.36^ab^

Note: compared with before treatment, ^a^*P* < 0.05. Compared with the control group, ^ab^*P* < 0.05.

**Table 4:** Comparison of clinical efficacy and complications between the two groups (*n* (%)).

Group	Get well	Get better	Invalid		Efficient
Control group (50)	24 (48.00)	14 (28.00)	12 (22.00)		38 (76.00)
Therapy group (50)	14 (28.00)	35 (70.00)	1 (2.00)		49 (98.00)
*χ* ^2^					10.698
*P*					0.001
Group	Skin rash	Chest tightness	Nausea	Diarrhea	Complication rate
Control group (50)	2 (4.00)	2 (4.00)	1 (2.00)	3 (6.00)	8 (16.00)
Therapy group (50)	0	1 (2.00)	0	1 (2.00)	2 (4.00)
*χ* ^2^					4.000
*P*					0.046

## Data Availability

No data were used to support this study.
